The article "Community matters: barriers and opportunities to sexual health and sexuality education of young female migrants in Hong Kong" was published in 2023. Journal: Front Psychol.

# Community matters: barriers and opportunities to sexual health and sexuality education of young female migrants in Hong Kong

**DOI:** 10.3389/fpsyg.2023.1270885

**Published:** 2023-11-27

**Authors:** Kim Kwok, Diana K. Kwok

**Affiliations:** ^1^Department of Social and Behavioral Sciences, City University of Hong Kong, Hong Kong, Hong Kong SAR, China; ^2^Department of Special Education and Counselling, The Education University of Hong Kong, Hong Kong, Hong Kong SAR, China

**Keywords:** community, sexual health, sexuality education, rights-based, young female migrants, structural vulnerability, sexual health model

## Abstract

**Introduction:**

Female migrant workers form a substantial portion of the global migrant workforce and research indicates they are vulnerable to sexual exploitation and barriers to sexual and reproductive healthcare. This article investigates the perceptions, barriers and opportunities to sexual health and sexuality education experienced by young female migrants in Hong Kong.

**Methods:**

The study adopted a rights-based perspective, employing qualitative methods for data collection, including focus group discussions and semi-structured interviews with 22 female migrants working as domestic workers.

**Results:**

Results indicate that young migrants’ perceptions of sexual health behaviors and access to sexuality education are shaped by various interconnected factors at four distinct levels: individual, interpersonal, social and community, and sociocultural and sociopolitical.

**Discussions:**

The present study adds to the existing literature by shedding light on certain perspectives that have not been given due emphasis in comparable studies. First, it highlights the importance of migrant community as barrier as well as opportunity in promoting positive health-seeking behaviors in a culturally acceptable manner. Second, it underscores the interplay between structural forces and individual and group-level vulnerability, emphasizing the need to address structural factors to eliminate young migrants’ internalized vulnerability. Third, it draws attention to the positive dimensions of sexual experiences as a motivator for proactive health-seeking and the intricate relationship between cultural practices and positive sexuality. This article recommends a proactive approach of migrant communities to address sexual healthcare issues while public healthcare institutions should proactively provide accessible sexual healthcare information and services.

## 1 Introduction

Sexual health is essential for lifelong wellbeing and includes respectful, positive and protected sexual experiences. The World Health Organization [WHO] (n.d.a) and scholars such as Sen (2014), Miller et al. (2015), and Gruskin et al. (2019) prioritize a human rights perspective, including rights to access to information and education, to maintain sexual health, to protect bodily autonomy and be free from sexual violence. Sexual and reproductive health is incorporated in the United Nations Agenda for Sustainable Development Goals (World Health Organization [WHO], n.d.b). Comprehensive sexuality education aims to provide non-judgmental information on a range of topics including gender norms and sexual expression to all young people following human rights principles (Berglas et al., 2014; UNESCO, 2018, 2021). However, traditional sexuality education based on Western theoretical constructs may not be effective for culturally diverse populations (Schmidt et al., 2012; Roodsaz, 2018). Culturally sensitive sexuality education has been recommended to acknowledge socio-cultural differences in sexual health perceptions and values, and to deliver messages in a culturally appropriate manner (Svensson et al., 2017; Szlachta and Champion, 2020; Kwok and Kwok, 2022).

Female migrant workers comprise a significant segment of the global migrant workforce. Specific challenges they encounter include vulnerability to sexual exploitation and barriers to sexual and reproductive healthcare (Keygnaert et al., 2014; Meldrum et al., 2016; Mengesha et al., 2017; Masuda et al., 2020). These stem from individual, group, and institutional factors, such as low awareness of sexual health, traditional beliefs about contraception, unfriendly staff attitudes as well as policy of migration regime that prioritizes cheap labor over protecting the labor and sexual rights (Webber et al., 2012; Ford and Holumyong, 2016; Boonchutima et al., 2017; Phanwichatkul et al., 2018; Masuda et al., 2020). Nevertheless, existing studies, particularly those in Asian context, have focused on a limited range of issues, such as HIV/AIDS, contraception, and unwanted pregnancies, overlooking important aspects of female migrant workers’ sexual health and sexuality education needs, such as emotional, mental, and social wellbeing related to sexuality and the positive and pleasurable dimensions of sexual experiences (Freeman et al., 2021). Although some studies address institutional and sociocultural factors, community-level factors have been largely neglected (Truong et al., 2014). Further exploration is needed to understand how migrant communities and organizations facilitate or hinder access to sexual health and sexuality education.

Hong Kong has around 350,000 migrant domestic workers, mostly Filipina and Indonesian women of childbearing age (Census and Statistics Department, 2022). Despite entitlement to a minimum wage, rest days, privacy, basic healthcare and pregnancy protection, these benefits are not always provided, rendering them vulnerable to exploitation (Amnesty International, 2013; Ullah, 2015; Paul and Neo, 2018). The power dynamics of their employment situation, negative stereotypes and racist depictions further exacerbate the vulnerability of female migrant domestic workers (Ladegaard, 2013; Olivotti, 2016). In view of these vulnerabilities and health and rights challenges, current research has investigated the mental health, COVID-related health, and the labor rights of migrant domestic workers in Hong Kong (e.g., Varia, 2011; Chung and Mak, 2020; Liem et al., 2021). However, sexual health remains under-researched, with only two studies on pregnancy rights (Paul and Neo, 2018; Constable, 2020).

This article examines the experiences of sexual health and sexuality education of young female migrants who worked as domestic workers in Hong Kong and identifies their barriers and opportunities. It employs a rights-based perspective to comprehend sexual health and sexuality education, and utilizes the concepts of structural vulnerability (Quesada et al., 2011; Truong et al., 2014) and the sexual health model (Tolman, 1999; Tolman et al., 2003) for analysis. Both frameworks offer appropriate lenses for this study, illuminating the gaps in previous research and outlining the implications for sexual health and sexuality education for this specific population.

## 2 Literature review

### 2.1 Rights-based sexual health

International scholarship has increasingly acknowledged sexual health as a fundamental human right. A rights-based approach has been employed (Sen, 2014; Miller et al., 2015; Gruskin et al., 2019) to better comprehend the availability of sexual healthcare. The World Health Organization has defined sexual health as “a state of physical, emotional, mental, and social wellbeing in relation to sexuality” (World Health Organization [WHO], n.d.a). This definition goes beyond the mere absence of dysfunction and disease and encompasses an attitude of respect and positivity toward sexuality and sexual relationships. It also includes the possibility of having consensual, non-exploitative and pleasurable sexual experiences that are protected against unintended pregnancy and sexually transmitted diseases (STDs). Various international agreements, including the World Conference on Human Rights of 1993, have outlined women’s rights to bodily autonomy and integrity concerning sexuality and reproduction, emphasizing that sexual violence violates human rights (Lottes, 2013). Scholars have therefore promoted a positive triangle of sexual health, sexual rights and sexual pleasure in law and advocacy (Gruskin et al., 2019). Significantly, sexual and reproductive health was included in the United Nations Agenda for Sustainable Development Goals in 2015, aimed at reducing health inequalities and achieving health equity (World Health Organization [WHO], n.d.b).

### 2.2 Comprehensive sexuality education in multicultural contexts

The comprehensive sexuality education model follows human rights principles and aims to provide accurate, non-judgmental information to all young people, regardless of their gender, sexual orientation, race, ethnicity, or gender expression (Berglas et al., 2014; UNESCO, 2018, 2021). This approach covers a broad range of topics, including gender norms, sexual expression, violence, and individual rights and responsibilities in relationships. Traditional sexuality education in Euro-American societies has been based on Western theoretical constructs and a worldview characterized by individualization and autonomy. However, this may not be effective for culturally diverse populations (Schmidt et al., 2012; Roodsaz, 2018). Scholars recommend culturally sensitive sexuality education that acknowledges the impact of cultural differences on health and sexual behavior (Svensson et al., 2017; Szlachta and Champion, 2020; Kwok and Kwok, 2022). Sexuality educators in multicultural contexts should be knowledgeable, comfortable discussing sensitive sexual issues, and aware of socio-cultural variations in sexual health perceptions (Szlachta and Champion, 2020). Sensitively addressing language and socio-cultural differences as well as conflicting sexual norms while emphasizing non-Western values like collectivism can promote a sense of unity and improve message adoption among culturally diverse learners (Svensson et al., 2017; Kwok and Kwok, 2022).

### 2.3 Female migrants’ sexual health and sexuality education

Despite its importance, female migrants in different parts of the world such as Europe (Keygnaert et al., 2014), Africa (Ivanova et al., 2018), and Australia (Meldrum et al., 2016; Mengesha et al., 2017) face inadequate sexual healthcare and sexuality education. Research in Asian context has concentrated on female migrant workers’ health risks and needs related to STDs (e.g., HIV/AIDs), contraception, unwanted pregnancies and need for safe abortion (Wong et al., 2012; Ayuttacorn et al., 2019; Masuda et al., 2020). For example, in Cambodia, female migrant workers expressed reluctance about modern contraception, leading to a higher risk of unintended pregnancy (Masuda et al., 2020).

The literature identifies individual, group, and institutional factors of sexual health access and sexuality education. At the individual and group levels, there are limited awareness of sexual and reproductive health, risky behaviors resulting from newfound freedom in a new environment, and traditional beliefs about contraception leading to infertility (Ford and Holumyong, 2016; Masuda et al., 2020). Additionally, due to cultural norms, some migrants fear sharing sexual health needs with family and community may lead to marital conflict, rejection, and loss of support (Ayuttacorn et al., 2019). At the macro level, institutional and policy constraints include high costs, inconvenient locations, long waiting times, unfriendly staff attitudes, and limited clinic hours (Webber et al., 2012; Boonchutima et al., 2017). Female migrant workers’ sexual healthcare and education are often not prioritized by their employers, industries, and national reproductive programs (Webber et al., 2010; Phanwichatkul et al., 2018). These could be attributed to receiving countries’ concerns about potential public health risks posed by migrant workers, prioritizing the supply of cheap labor over protecting these workers’ labor and sexual rights (Truong et al., 2014; Piper et al., 2017).

The above review highlights that existing studies on female migrant workers’ sexual healthcare and sexuality education in Asian context focus overwhelmingly on a limited range of issues, such as HIV/AIDS, contraception and unwanted pregnancies, possibly due to the public health discourse of the receiving country prioritizing the absence of dysfunction and disease (Freeman et al., 2021). This focus has resulted in the neglect of critical aspects of young female migrants’ sexual health needs and education, such as sexual expression, pleasurable aspects of sexual experiences, emotional and social wellbeing regarding sexuality, violence and gender norms. Although several studies have examined institutional, policy, and sociocultural factors (e.g., Webber et al., 2012; Phanwichatkul et al., 2018; Masuda et al., 2020), community-level contexts have received less attention (Truong et al., 2014). There has been little exploration of how migrant communities and organizations facilitate or impede access to sexual healthcare and sexuality education.

### 2.4 Migrant domestic workers’ structural vulnerability in Hong Kong

Scholars have advanced the concept of structural vulnerability to explain health inequality and ill health (Quesada et al., 2011). The concept pertains to the position of individuals within the social hierarchy, which imposes limitations on or enhances their capacity to contest and negotiate power dynamics that impact their health. It goes beyond the binary distinction between structure and agency and addresses the interplay between the objective (structural forces) and the subjective (individual perceptions and will). According to Truong et al. (2014), migrant domestic workers’ vulnerability can be understood as resulting from multiple institutional discriminations (migrant status, ethnicity, gender, age, etc.), intersecting with the labor migration and healthcare systems.

Hong Kong has recruited migrant domestic workers since the 1970s. Currently, there are approximately 350,000 in the territory, most of whom are women of childbearing age, with almost equal proportions from the Philippines and Indonesia and smaller numbers from Thailand, India, Nepal, and Bangladesh (Census and Statistics Department, 2022). Migrant domestic workers in Hong Kong are subject to a 2-year employment contract regulating their wages, rest days, mandating their residence with their employer and prohibiting them from engaging in any paid work other than domestic work. Despite being entitled to a minimum wage, rest days, privacy, basic healthcare, and pregnancy protection, research shows that migrant domestic workers cannot always access these benefits, leaving them susceptible to exploitation and abuse (Amnesty International, 2013; Ullah, 2015; Paul and Neo, 2018). For example, they are entitled to public medical services; however, their access may be curtailed if their employer restricts their mobility beyond Sundays, when many public services are closed. The power dynamics of the domestic work setting, where the legal status and employment of migrant workers are contingent on their employer, create an asymmetrical power relationship exacerbating domestic workers’ existing vulnerability. Additionally, female migrant domestic workers are often subject to negative stereotypes and racist depictions in popular discourses, portraying them as culturally inferior and morally suspicious “racialized others” (Ladegaard, 2013; Olivotti, 2016). As such, the convergence of government regulations, the nature of migrant domestic workers’ work, migrant status, gender and ethnicity positions them at the bottom of the social hierarchy, resulting in structural vulnerability that shapes their healthcare, health-seeking behaviors as well as access to health education. One impact is a fear of asserting their pregnancy protection rights (Paul and Neo, 2018). Given their structural vulnerability, a substantial body of research has investigated their various health and rights challenges such as mental health, COVID-related health, and labor rights (e.g., Varia, 2011; Chung and Mak, 2020; Liem et al., 2021). However, except two studies on pregnancy rights (Paul and Neo, 2018; Constable, 2020), relevant research on sexual health and sexuality education among this population remains scant.

## 3 Materials and methods

This study utilized a qualitative descriptive approach (Braun and Clarke, 2006; Nicholas et al., 2013) to investigate the experiences of young female migrant workers in Hong Kong regarding their sexual healthcare and sexuality education. This approach allows for “identifying observations and constructs emerging from narrative-based data” without adopting a specific theoretical lens (Nicholas et al., 2013, p. 867). Besides, this study combined focus group and individual interviews for data triangulation to enhance data richness (Carter et al., 2014).

### 3.1 Data collection and participants

Before collecting data, ethical approval from the Education University of Hong Kong (Ref. 2019-2020-0245) was obtained. The research participants were informed about the study’s purpose, data usage, their right to decline answering questions or withdraw from the interview, and the confidentiality of the study. Consent was obtained from all participants before interview and discussion took place. Purposive sampling was used to recruit participants through informal and formal connections, such as support groups and NGOs providing HIV tests and services for pregnant migrant workers. Inclusion criteria for participation were: (1) being a female migrant domestic worker in Hong Kong, and (2) having experiences of utilizing/needing sexual healthcare and relevant information in Hong Kong. Twenty-two young women participated in this study, ranging in age from 22 to 36 with an average age of 28.2. All were born outside Hong Kong with an average residence duration of 3.1 years in Hong Kong. They participated in two Zoom focus groups, one with Indonesian (*n* = 6) and one with Filipina participants (*n* = 6), and subsequent semi-structured individual interviews with six Indonesians and four Filipinas. Saturation of data was checked by employing the code meaning strategy (Hennink and Kaiser, 2022).

The focus groups facilitated an initial understanding of our target participants’ perceptions of the topic. Relatively non-sensitive issues were raised and discussed that included sexuality education in home country, information about sexual health and reactions in the migrant communities in Hong Kong, and protection against sexual harassment in their work place. Based on the focus group discussions, a semi-structured interview guide was then prepared and inductively refined on the basis of emerging themes throughout the interview process. It included questions about participants’ sexual health selfcare, knowledge and awareness, information and healthcare access, contraception, negotiation in intimate relationships, HIV testing, resources and constraints in the work environment, risk of sexual harassment, and community resources and constraints. The semi-structured individual interviews explored individual experiences in depth. They were held in mutually agreed venues, either at NGOs or other locations chosen by the participants. Two were conducted through Zoom. Most interviews were conducted in English or Cantonese, while the Indonesian focus group discussions were conducted in Bahasa Indonesia with the assistance of a community interpreter. Additionally, two NGO workers with experience in providing sexual and reproductive health services for female domestic workers were interviewed.

The researchers employed various techniques such as bracketing and presuppositions before, during, and after data collection to minimize subjectivity. The researchers disclosed their own backgrounds, remained receptive to understanding participants’ perceptions, and shared relevant personal experiences to mitigate power imbalances between the researchers and study participants and between the cultural majority and minority groups. The interviews were conducted collaboratively using open-ended questions, such as “please share your experiences of learning sexual and reproductive healthcare information in Hong Kong.” The researchers used semi-structured questions to alleviate unease when any participant exhibited discomfort with open-ended questions. Individual interviews were audio recorded and transcribed, and researchers’ field notes were used to record focus group discussions. All names used in this article are pseudonyms to protect participants’ confidentiality.

### 3.2 Data analysis

The data were analyzed following Braun and Clarke’s (2006) five-step qualitative thematic analysis approach. Firstly, the research team acquainted itself with the data by repeatedly reading the interview transcripts and field notes. Second, the team generated initial codes such as body knowledge, trust in monogamy and partners, exploration in sexuality, and sexual harassment. Third, through discussion, the team organized the codes, leading to the emergence of themes with relevant data extracts such as “personal beliefs,” “accommodating intimate partners,” “community silence,” and “lack of institutional support.” Fourth, the coded themes were revisited and assessed for coherence. Finally, the emergent themes were refined and overarching themes identified. The finalized codes were agreed upon by the research team.

During this final phase, the sexual health model (Tolman, 1999; Tolman et al., 2003) was employed to identify and analyze the factors influencing the sexual healthcare and information access of migrant workers at the individual, interpersonal, social and community relationship and sociocultural and sociopolitical levels. The sexual health model integrates feminist, relational, and ecological theories and places individuals in social contexts and considers institutional, cultural, and policy factors that impact individuals. This model is distinctive because it goes beyond material resources such as contraception and includes information on sexual expression and alternative discourses such as female sexuality besides sexual intercourse. This model addresses patriarchal ideologies that limit female sexuality and pleasurable relationships, while also questioning power and privilege. The framework includes four interplaying contexts, (1) individual women’s practices, knowledge, attitudes, and values toward sexual health, (2) the interpersonal context of romantic relationships, including expression of sexual desire and making active choices, (3) social relationships affecting sexual health, including support in working through confusions, and (4) sociocultural and sociopolitical contexts, including access to and freedom to use sexual and reproductive healthcare. The sexual health model is relevant to this study, with two main observations justifying its use. First, young migrant domestic workers’ engagement with sexual and healthcare and sexuality education is affected by various factors, and there are dynamic interrelationships between the migrants and their social environments, including their interpersonal contexts and migrant worker communities. The sexual health framework can comprehensively acknowledge the many factors involved and propose targeted enhancement strategies. Second, despite facing structural vulnerability and patriarchal norms, some young migrant workers did engage in sexual expression and sexual healthcare behaviors that are different from the conventional feminine ones. Application of the sexual health model can elucidate the influence of patriarchal power on women’s sexuality while also revealing opposing forces.

This process enabled the researchers to identify unique stories and arguments of this study (see Table 1). Some participants and community interpreters were provided with the preliminary findings and analysis to ensure the study’s trustworthiness.

**TABLE 1:** Themes and overarching themes of data.

Individual	Interpersonal	Social and community	Sociocultural and sociopolitical
● Inadequate knowledge ● Personal beliefs	● Accommodating intimate partners ● Breaking with social conventions ● Avoiding reporting health issues ● Vulnerability to sexual harassment	● Community’s relative silence ● Community pressure	● Lack of institutional support and accepting services ● Discouraging societal attitudes

## 4 Results

Results are categorized into four levels: individual, interpersonal, social and community, and sociocultural and sociopolitical.

### 4.1 Individual level

#### 4.1.1 Inadequate knowledge

Participants revealed inadequate biological understanding, including menstruation and pregnancy, one possible reason hindering their ability to take adequate care of themselves, especially among Indonesian participants. For example, Gina had never touched a condom in her life. Her response to being asked if she knew how a baby is produced, was:

it comes naturally …It’s like a secret. We didn’t talk about it openly. We just learn by situation …In Indonesia, they tell children that when you have blood in your vagina, it means you have grown up, be more careful, don’t let any men touch you as it may get you pregnant … there is no education as to why you become pregnant, how you can prevent pregnancy with your husband.

Other participants from Indonesia shared similar stories about their experiences. One even recalled how she was taken aback when having her first period because her parents did not prepare her for it. Instead, they only taught her how to be a good wife to her future husband.

#### 4.1.2 Personal beliefs

Beliefs about menstruation, condom use, HIV testing and women’s role in sex inhibited participants from safeguarding themselves. For instance, Gina demonstrated her firmly held perception that protection was unnecessary for someone in a trustworthy monogamous relationship: “For me, those who are honest with their husbands wouldn’t need it [condom and HIV test].” Participants shared that in Java, it is believed that sex is primarily for men while women would become stronger after giving birth. Therefore, it is a tradition not to use condoms in order to increase the likelihood of giving birth.

Some participants actualized their beliefs in practice at the expense of personal hygiene:

When we [in Indonesia] are menstruating, we do not shower, [even] if we shower, we do not wash our hair. … I shower but do not wash hair …[because] it is very uncomfortable here in Hong Kong, especially in summer, after working in the kitchen … [we believe otherwise] this will harm your body (Teresa, Indonesian).

There appears to be a potential linkage between inadequate knowledge and deeply ingrained beliefs, such as a trustworthy relationship does not need protection and sex is men’s domain, which participants’ cultural upbringing could shape. The latter served as justifications that limited participants to seek more explanation through education and access to information and maintain their reproductive health through necessary hygiene practices.

### 4.2 Interpersonal level

#### 4.2.1 Accommodating intimate partners

Intimate relationships and interactions with partners generated concerns about sexual health. For instance, participants often accommodated or acquiesced to their male partner’s wishes not to use a condom even though they knew condom use offered protection from STDs. This may be linked to the perception that sexuality is primarily a male domain. Isa (Filipina), referred to not using a condom:

He [my boyfriend] is not using it … he does not like to use … I know the good thing [about using condom] is that you’re protected from disease, I never think of this [STD can happen to me].

Some participants struggled to comply with their boyfriend’s wishes before ultimately giving in. Maria (Filipina) recalled: “I was not sure, I struggled, because it was in my time, growing up in the Philippines, not common to use condom … but my British boyfriend insisted on using a condom…”

#### 4.2.2 Breaking with social conventions

Working far from home, some participants experienced their husband’s infidelity, prompting them to change their attitudes and behavior. Erina (Filipina) recounted that condom use and HIV checks are uncommon for migrant workers; however, she broke with the social convention: “… my husband cheated on me, so I did the [HIV] test to make sure I was fine, even if my people judge me negatively.”

Working outside their home country provided the opportunity and freedom to explore female sexuality and pay attention to safe sex practices, which would have otherwise been impossible. Srina (Indonesian) described her experience:

Before I came to Hong Kong I usually had a boyfriend. When I came to Hong Kong, I started having sex with women … I first met someone at the training center in Surabaya, she was a tomboy, felt comfortable with her. It was my first time feeling connected and attracted. but my family is conservative, [I could] never imagine this before … we discussed protection, we try to find solutions [on internet] to have safe sex…. With women I am happier in sex.

#### 4.2.3 Avoiding reporting health issues

Requirements to live in their employer’s household strongly impacted young migrant workers’ sexual healthcare and information access. Our participants often avoided reporting health issues to their employers and seeking help from them because they worried they would be blamed for not avoiding the problem. Eighteen participants had never undergone a general gynecological check-up or pap smear test. If they felt ill during their period, they carried on working as normal. Their usual “cure” was to take painkillers. Even though entitled to basic medical care, many were ill-informed of their rights and scared to ask for time off for a medical appointment:

They [employers] blame you before giving you help. That’s why I cure myself, not let them blame you … when I was stressed at work, my period was late, and when it came, it was so heavy, so full, that I really felt sick … never thought of going to see a doctor (Davina, Filipina).

#### 4.2.4 Vulnerability to sexual harassment

Migrant workers were vulnerable to sexual harassment in their employer’s household. They felt they could not challenge or clarify ambivalent situations but had to tolerate them to keep their jobs. Several mentioned being groped by male employers or the employer’s relatives. Female employers were usually unaware of these instances and participants were afraid to tell them: “I did not tell her because I am afraid she would not believe me,” said Lila (Filipina). Gina described an ambivalent situation that embarrassed her: “the son of the family always walks around in the apartment in his underwear. He is over 20. … I feel strange and uncomfortable. But what shall I say?”

### 4.3 Social and community level

#### 4.3.1 Community’s relative silence

Participants observed that their communities considered discussions of sex and intimate relationships taboo, resulting in a culture of silence. Therefore, little useful information or assistance could be sought. For example, Davina reported her experience in the church:

I mostly spend Sundays in church. For them, if you try to open that [sex] issue, it’s too malicious, too vulgar … my churchmates are afraid. When we started to talk about sex, they tried to change the topic … I tried to ask them about their boyfriends, their lives, if they kiss … They did not want to answer me.

Srina joined a local NGO as a community ambassador to promote sexual health and rights knowledge to fellow Indonesian migrant workers. She revealed that she encountered great difficulty in spreading the message. Some fellow migrant workers rejected her by saying “we don’t want to know about this.” Although numerous migrant associations deal with various concerns of domestic workers, sexual healthcare issues are not well-addressed. Less effort had been put into awareness-raising and information dissemination. Srina noticed: “they [migrant associations] care about our work problems, contract problems … but no one [in the migrant associations] tells us what to do when we are pregnant, where to ask for help for body check-up….”

Despite this, one Indonesian participant recollected a past instance in which a religious organization had hosted an educational session on sexual health that attracted a notable level of attendance. However, such occurrences were not commonplace.

#### 4.3.2 Community pressure

Respondents reported feeling pressure from their community. Many were afraid that their identity would be exposed if they openly went for HIV testing. The relative silence and pressure surrounding sexual topics might result from cultural assumptions, such as the belief that women who go for HIV testing are “promiscuous” or engage in multiple casual sexual relationships, implying that only such women are at risk of contracting HIV. Hana (Indonesian) echoed Gina’s belief but applied it to the community level:

Most people in the Indonesian community in Hong Kong do not care about HIV. I asked many friends to come for testing, but they refused; public education [in our community] is not enough …People think that once you are married, this HIV thing is not an issue anymore.

### 4.4 Sociocultural and sociopolitical level

#### 4.4.1 Lack of institutional support and accepting services

One frequently mentioned barrier to sexual healthcare was the unfriendly attitude of some healthcare and service institutions. For example, Hong Kong Family Planning Association (FPAHK), a government-funded organization promoting sexual health and rights and providing services such as pregnancy check-ups and birth control services, failed to offer the same services and relevant education to migrant domestic workers. Inconvenient service hours and information about services overlooked the potential for negative labeling, as recounted by Jasmin (Filipina):

I remember I read their promotion materials, but they are closed on Sunday … Later, on Sunday, they organized a van, it was mobile service, they made everything in a van, but no one dares to go, people do not want to be seen going to the van.

While promotion materials were printed in various languages including Bahasa Indonesian apart from English and Chinese, the FPAHK website provided only English and Chinese information.

Siti (Indonesian) recalled her experience of seeking help and consultation regarding sexual harassment:

Last year my cousin’s new employer touched her, and made [a sexual] quest again and again … she was frustrated and depressed. I asked my Chinese friend to help, and she called everywhere … no service [organization] could help, because they all work from Monday to Saturday. No one works on Sunday … She left the job.

Sandra (Chinese), working for the sole NGO in Hong Kong offering services to pregnant migrant women and promoting their sexual healthcare, highlighted another instance of institutional neglect. Her NGO received no regular public funding: “we have only short-term and project-based funds. But we are helping the women and their babies, this cannot be project-based.”

#### 4.4.2 Discouraging societal attitudes

Prevailing societal attitudes in Hong Kong discourage migrant workers from seeking sexual health information and assistance and suggest that migrant workers are responsible for working diligently and staying fit for work, instead of enjoying their rights to sexual and reproductive healthcare. As Davina commented, employers usually expect them to be accountable for staying healthy: “They [employers] blame you before giving you help, that’s why I cure myself, not let them blame you.”

According to Sandra, a significant number of Hong Kong people, particularly employers, believe migrant domestic workers are not entitled to pregnancy-related healthcare. This led to the perception that terminating the employment of a pregnant migrant worker was legally acceptable:

In Hong Kong, the law [Employment Ordinance] provides maternity protection and healthcare to all women, migrant domestic workers, too… but some employers still ask their pregnant workers to abort, or they dismiss them.

## 5 Discussion and implications

### 5.1 Community matters: a site where barriers and opportunities coexist

Migrant community matters in promoting sexual health and providing sexuality education for migrant workers because it represents a site where not only barriers are present, but also opportunities. Despite being cognizant of the potential pitfalls of communities, their role remains crucial due to the efficacy of culturally appropriate and reliable community-based educational initiatives (Gosselin et al., 2019; Hawkey et al., 2022). However, this study reveals that the relative silence within migrant domestic worker communities in Hong Kong impedes the promotion of sexual health and sexuality education. This may be due to the passive stance of migrant organizations toward community education on this topic, leading to pressure on individual migrant workers, as shown in the study. Hong Kong is home to numerous organizations catering to migrant domestic workers, but their exact number is difficult to ascertain. As this study’s participants highlight, little community public education addresses sexual health issues. Many organizations are preoccupied with labor issues and a few faith-based associations actively assist abuse victims. As a result, sexual health concerns and sexuality education are easily overshadowed (Truong et al., 2014).

Apart from barriers, opportunities also exist, as suggested by our findings, such as the well-attended information session hosted by an Indonesian religious organization. Communities provide not only valuable networks and resources, but also cultural familiarity and a relatively trustworthy environment in which young migrants workers feel more comfortable sharing and receiving information (Svensson et al., 2017; Szlachta and Champion, 2020; Kwok and Kwok, 2022).

Therefore, this study recommends a more proactive approach from migrant domestic worker communities, community leaders, volunteers, bicultural workers, and religious organizations to address the issue. They are in a favorable position to raise awareness, promote positive health-seeking behavior, dispel myths, and clarify beliefs (such as the misconception that getting an HIV test implies a lack of sexual fidelity) in a culturally sensitive manner. For instance, when introducing sexual rights and pleasure, migrant community educators can better address some cultural values relevant to the particular community, such as collectivism. Besides, mainstream sexual healthcare institutions should collaborate with domestic worker community organizations and charities to augment community education on this issue. Public funding should be offered to encourage such educational activities.

### 5.2 Structural vulnerability: mutual influence of multiple barriers

The use of the concept of structural vulnerability offers insights for this study. First, it helps explain how multiple structural forces, such as legal conditions, socioeconomic status, gender, ethnicity, and cultural norms, intersect to create a type of structural violence that disadvantages young migrant workers, denying them access to sexual health and sexuality education. This phenomenon is observable in various contexts of participants’ lives, such as limited knowledge and deep-seated beliefs about female sexuality influenced by cultural norms imbued with patriarchal values (e.g., sex is men’s domain) in broader sociocultural contexts (Medina, 2008; Riyani and Parker, 2018). These factors generally reduce their negotiating ability in intimate relationships to safeguard their sexual health and motivation to seek for relevant information at the interpersonal level. Second, the concept of structural vulnerability highlights the perspective of young female migrant workers who mostly do not perceive themselves as having the right or ability to assert their sexual health and sexuality education. Although participants were not explicitly informed about their entitlement or denial of sexual healthcare and sexuality education, institutional neglect, discrimination by employers, and discouraging attitudes of the general public created a barrier to contesting discrimination and exclusion. Consequently, they passively accepted and internalized their vulnerability, disengaging from their sexual healthcare and help seeking. This led to refraining from pregnancy protection (Paul and Neo, 2018) and underreporting of harassment and abuse due to fears of losing their job and residency in Hong Kong (Equal Opportunity Commission, 2014; Ullah, 2015).

As such, it can be posited that the barriers encountered across diverse contexts demonstrate a mutual influence or reinforcement. This has implication for sexual health and sexuality education in practice. In addition to public education to raise awareness of rights among employers and migrant workers, institutional neglect and discouraging societal attitudes should be tackled to alleviate internalized vulnerability. Without addressing internalized vulnerability, migrant workers may be disinclined to assert their rights and seize opportunities proactively. We therefore recommend public healthcare institutions in receiving countries provide accessible services and information to migrant workers, including alternative modes of service delivery, flexible service hours and information in readily understandable language for migrant workers. Sending countries should provide pre-migration training to clarify migrant workers’ sexual health rights. These institutional and sociocultural measures should gradually enhance individual, interpersonal and community-level capabilities to protect and negotiate for sexual health rights.

### 5.3 Agency for positive sexuality and health-seeking

While the findings of this study suggest that patriarchal norms impact the sexual perceptions and behaviors of young female migrant workers, some participants demonstrated agency in challenging conventional sexual practices. For instance, some participants who had experienced infidelity were more willing to engage in protective measures, such as undergoing HIV testing. Being far from home, these migrants were relatively free to explore alternative sexuality, such as same-sex desire offering a sense of attachment and sexual pleasure, in turn motivating them to safer sexual health practice. Notably, the opportunity for exercising agency and positive sexuality occurred within the context of migration. Although existing literature suggests the linkage between migration and sexual freedom (e.g., Hoy, 2007), determining whether this migration context fosters such agency is challenging because of the lack of adequate data. Nevertheless, these results suggest that sexuality is not solely a site of control and oppression, but also a realm of pleasure and emancipation. Furthermore, it is important to note that traditional cultural norms and practices pertaining to sexual matters are not fixed, but rather dynamic and susceptible to environmental factors, such as the experience of migration. This highlights the intricate interplay between cultural beliefs and practices and positive sexuality.

Thus, the study reiterates the importance of understanding sexual health and sexuality education beyond the absence of dysfunction and disease, as emotions and pleasure are significant components of female sexuality that can motivate women to pursue sexual health and are integral to their sexual rights (World Health Organization [WHO], n.d.a). However, the literature on sexual healthcare interventions and promotion seldom mentions these positive aspects, possibly due to their sensitive nature, particularly in certain cultural contexts such as Asia (Woo et al., 2011; Riyani and Parker, 2018). This prompts us to re-emphasize the need for culturally sensitive approaches to address sexual health and rights in a trustworthy environment (Svensson et al., 2017; Szlachta and Champion, 2020; Kwok and Kwok, 2022).

## 6 Conclusion

This paper contributes to research on sexual health and sexuality education of young migrant workers. First, the application of the concept of structural vulnerability highlights the interplay between structural forces and individual and group-level vulnerability, which illustrates how barriers encountered across various contexts exhibit a reciprocal influence or reinforcing effect. This approach has practical implications for addressing the issue, suggesting that public education efforts alone may be insufficient to overcome internalized challenges experienced by migrant workers. Efforts to address structural factors, such as institutional neglect and negative societal attitudes, are also necessary. Second, this study emphasizes the significance of migrant worker community as barrier and opportunity in raising awareness, addressing sexual health challenges, promoting positive health-seeking behavior, and dispelling myths. Collaboration between mainstream healthcare institutions and community organizations is necessary, with public funding to support educational activities. Third, the study draws particular attention to the positive dimensions of sexual experiences, such as pleasure, intimacy, and emotional bondage, as a motivator for proactive health-seeking. Additionally, it underscores the intricate relationship between cultural beliefs and practices and positive sexuality. Implication is that there is a need for cultural sensitivity and a trustworthy environment such as the migrant community to effectively improve the sexual health awareness and outcomes of migrant workers in the Asian context. These perspectives are valuable in advancing our understanding of sexual health and sexuality education of female migrant workers, as they have not been previously emphasized in similar studies.

The study has limitations. First, participants were recruited through purposive sampling, so might have been more willing to discuss and contemplate their experiences than others. Nevertheless, cultural constraints may have increased participants’ reluctance to share their experiences thoroughly. Therefore, caution should be exercised in generalizing the findings to other contexts. Second, the study did not distinguish between Indonesians and Filipinas; their diverse cultural backgrounds, religious beliefs, and linguistic abilities may have varying effects on their sexual healthcare and sexuality education experiences. Thus, future research could be improved by examining the differences among specific groups of migrant workers. Third, due to time constraint, this study was not able to include a broader group of stakeholders including healthcare workers. This may affect the depth of our understanding of the problem.

## Data availability statement

The datasets presented in this article are not readily available due to confidentiality, only part of the dataset can be assessed upon request. Requests to access the datasets should be directed to KK, kimkwok@cityu.edu.hk.

## Ethics statement

The studies involving humans were approved by the Human Research Ethics Committee, the Education University of Hong Kong. The studies were conducted in accordance with the local legislation and institutional requirements. The participants provided their written informed consent to participate in this study. Written informed consent was obtained from the individual(s) for the publication of any potentially identifiable images or data included in this article.

## Author contributions

KK: Conceptualization, Data curation, Formal analysis, Investigation, Methodology, Project administration, Writing – original draft, Writing – review and editing. DK: Conceptualization, Methodology, Writing – review and editing.
